# Clinicopathological Characteristics and Prognostic Factors of Primary Bladder Signet Ring Cell Carcinoma

**DOI:** 10.1155/2022/3224616

**Published:** 2022-09-05

**Authors:** Liang Liu, Qiang Wang, Haibo Yuan

**Affiliations:** Department of Urology, Baoding No. 1 Central Hospital, Baoding 071000, Hebei, China

## Abstract

**Introduction:**

The aim of this study is to examine the treatment pattern and predictors of long-term survival of patients with primary signet ring cell carcinoma (PSRCC) of the urinary bladder based on the analysis of the SEER database.

**Methods:**

The 3-year and 5-year overall survival (OS) and cancer-specific survival (CSS) were calculated using the Kaplan–Meier method. Then, we compared the CSS curves by the log-rank test. The independent risk factors were determined using univariate and multivariate Cox regression.

**Results:**

The 3-year OS and CSS rates for PSRCC of the bladder were 25.3% and 33.3%. The 5-year OS and CSS rates for the entire cohort were 16.4% and 25.2%. The CSS rates, respectively, were 0, 25.0, 66.7, 33.2, 42.4, and 31.7% at 3 years and 0, 25.0, 34.3, 24.1, 27.2, and 31.7% at 5 years for none, transurethral resection of the bladder (TURB), partial cystectomy, radical cystectomy with reconstruction, pelvic exenteration, and other surgeries (*P* = 0.001). Multivariate analyses showed independent risk factors only including T stage, M stage, lymph node removal, and surgical approach.

**Conclusions:**

T stage, M stage, lymph node removal, and surgical approach are independent risk factors of PSRCC of the urinary bladder. TURB and radical cystectomy with reconstruction appear to provide a better outcome.

## 1. Introduction

Bladder tumor is one of the most common malignancies and among the most prevalent causes of tumor-associated deaths over the world. According to reports, there are more than 300,000 patients diagnosed with bladder cancer each year and more than 165,000 patients died each year [1, 2]. Primary signet ring cell carcinoma (PSRCC) of the bladder, a rare type of a bladder tumor, is accounting for approximately 0.12%–0.6% of all bladder malignancies [3, 4]. PSRCC, classified as a subtype of bladder adenocarcinoma, has the worst prognosis [5, 6]. However, according to the World Health Organization classification in 2016 for tumors of the urinary system and male genital organs, PSRCC belongs to the subtype of invasive urothelial carcinoma [7]. Patients are usually around 60 years, and the male/female ratio is about 3 : 1 [8, 9]. Similar to bladder urothelial carcinoma, the most familiar symptoms are hematuria in 65% of cases, which are usually painless [10]. However, the clinical manifestation is nonspecific, which leads to the patients having already reached an advanced stage and with a poor prognosis.

A standardized treatment protocol for the treatment of PSRCC has not yet been founded, and surgery is the main mode of treatment, but there is no consensus on the surgical modalities. Despite PSRCC being highly malignant, it is often ignored by clinicians due to its less incidence. For these purposes, we analyzed data on PSRCC of urinary bladder patients by the national Surveillance, Epidemiology, and End Results (SEER) database between 2004 and 2015. Meanwhile, we also explored the prognostic values of the clinicopathological features and survival outcomes.

## 2. Materials and Methods

### 2.1. Data Sources and Variables

Data from the NCI SEER program, collected from 2004 to 2015, were retrospectively analyzed. SEER*∗*Stat (Surveillance Research Program, National Cancer Institute SEER*∗*Stat software, version 8.3.8) was used to extract case-level data.

Inclusion criteria were as follows: (1) age≥ 20 years; (2) the primary site was restricted to the urinary bladder (C67.0–C67.9) according to the ICD-O-3; (3) histology only included SRCC (ICD-O-3 8490/3); (4) confirmed by positive histology and the first positive indicator of malignancy; (5) staging was according to the 6th edition of the American Joint Committee on Cancer (AJCC) Staging Manual. Exclusion criteria were as follows: (1) without histological diagnosis; (2) without survival data; (3) histological grade or AJCC stage information was unknown; (4) the scope of regional lymph node surgery was unknown.

Patient demographics analysis included gender, age, race, and year of diagnosis. Tumor characteristics studies included tumor size, AJCC 6th stage group, T stage, N stage, M stage, and histologic grade. Treatment characteristics included surgery and lymph nodes removal.

### 2.2. Statistical Analysis

All data were analyzed by SPSS software version 25.0. The 3-year and 5-year overall survival (OS) and cancer-specific survival (CSS) were calculated using the Kaplan–Meier method. The overall survival curves and cancer-specific survival curves were plotted according to the Kaplan–Meier method and compared with the cancer-specific survival curves by the log-rank test. The independent risk factors of SRCC were determined using univariate and multivariate Cox regression. *P* < 0.05 was considered statistically significant.

## 3. Results

### 3.1. Demographics and Tumor Characteristics

Table 1 lists the demographic and pathological characteristics of the PSRCC patients.

### 3.2. Survival Outcomes

The 3-year OS and CSS rates for PSRCC of the bladder were 25.3% and 33.3%. The 5-year OS and CSS rates for the entire cohort were 16.4% and 25.2% (Figures 1(a), 1(b)).  Figure 2 shows the survival estimates stratified by AJCC stage, N stage, M stage, tumor size, surgery status, and lymph nodes removed. The CSS rates, respectively, were 0, 25.0, 66.7, 33.2, 42.4, and 31.7% at 3 years and 0, 25.0, 34.3, 24.1, 27.2, and 31.7% at 5 years for none, transurethral resection of the bladder (TURB), partial cystectomy, radical cystectomy with reconstruction, pelvic exenteration, and other surgeries (Figure 2(e)). The 3-year and 5-year CSS rates for patients who had not lymph nodes removed were 27.5 and 21.8%, removed 1 to 3 regional lymph nodes all were 0%, and removed 4 or more regional lymph nodes were 41.2 and 30.6%, respectively (Figure 2(f)).

### 3.3. Prognostic Factor Analysis

In this study, univariate analyses confirmed that risk factors of PSRCC of the bladder include tumor size, M stage, lymph node removed, and surgical approach. However, multivariate analyses showed that independent risk factors only include T stage (T3 vs. T1, HR = 4.306, 95%CI = 1.770–10.478, *P* = 0.001, T4 vs. T1, HR = 2.765, 95%CI = 1.218–6.277, *P* = 0.015), M stage (HR = 2.343, 95%CI = 1.334–4.118, *P* = 0.003), lymph node removed (4 or more regional vs. none, HR = 0.477, 95%CI = 0.247–0.922, *P* = 0.028), and surgical approach (TURB vs. none, HR = 0.255, 95%CI = 0.109–0.601, *P* = 0.002; partial cystectomy vs. none, HR = 0.125, 95%CI = 0.040–0.389, *P* < 0.001; radical cystectomy with reconstruction vs. none, HR = 0.193, 95%CI = 0.080–0.467, *P* < 0.001; pelvic exenteration vs. none, HR = 0.132, 95%CI = 0.049–0.354, *P* < 0.001; and other vs. none, HR = 0.129, 95%CI = 0.039–0.424, *P* = 0.001) (Table 2).

## 4. Discussion

In this study, we aimed to discuss the prognostic value of the clinicopathological characteristics and survival outcomes in PSRCC of the urinary bladder.

PSRCC of the urinary bladder is a rare bladder malignancy, which belongs to the subtype of invasive urothelial carcinoma, with a lower incidence rate [7]. Holmäng et al. [11] reported that PSRCC of the bladder patient's occupancy 0.6% in 713 bladder cancer patients. PSRCC of the bladder was less commonly reported since the first patient was reported by Saphir [12]. Most studies were case reports, single-center studies, or small sample studies, but few researchers have analyzed the prognostic factors involved [13–17].

In this study, 106 (67.5%) patients were AJCC stage III or IV, and 49 (31.2%) patients were grade IV at diagnosis in our study, which indicates that PSRCC has the characteristics of a highly invasive and poorer prognosis. Our study agrees with the study by Akamatsu et al. [9]. In their study, the higher the histological grade, the worse the clinical prognosis (2-year OS, 43%). Besides, 46% patients were AJCC IV stage, and the survival time was not more than 2 years. The present study revealed that 62.4% patients had no lymph node metastasis and 82.8% patients had no distant metastasis. Although the PSRCC of the bladder had a lower rate of lymph node metastases and distant metastases, their prognoses were worse. According to the literature reported, the survival rate of PSRCC was lower than that of bladder urothelial carcinoma, and the natural course of the disease was 3.5 months [18]. The 5-year OS rates in our study for AJCC stages II, III, and IV were lower than those in the previous study (34.7% vs. 75%, 16.4% vs. 38%, and 6.0% vs. 12%)[10]. A Japanese study reported by Dadhania et al. [19] also demonstrated that almost half of the PSRCC patients were already at AJCC stage IV at the time of diagnosis, and the median survival was about 8 months. Besides, the surviving period of time did not exceed 2 years. However, the 5-year survival rates were nearly 50% for stages I–III in SRCC of the bladder. In our cohort, 73 (46.5%) patients were AJCC stage IV, the median survival time was 13 months, and the maximum survival time was 162 months. In addition, one study based on the SEER data in the US showed that 3-year CSS was 32% for PSRCC of the bladder, which was in accordance with our study (3-year CSS 33.3%) [18]. However, 3-year CSS was 67% of bladder urothelial carcinoma. It indicates worse outcomes for patients with bladder urothelial carcinoma than PSRCC.

Simultaneously, compared with OS curves and CSS curves, Kaplan–Meier survival curves are close (Figures 1(a), 1(b)). The common feature suggests the majority of the deaths were from SRCC causes. They further showed its poor prognosis characteristics. In our study, the 3-year OS and CSS rates for primary SRCC of the bladder were 25.3% and 33.3%. The 5-year OS and CSS rates for the entire cohort were 16.4% and 25.2%. The results were consistent with those of Wang et al. [20] (3-year CSS 40.6%), and they found that 60%–70% patients die within three years due to PSRCC of the bladder.

As for the PSRCC of the bladder, there have been differences among clinical study results of the prognostic factors for survival.

Multiple studies, compared with PSRCC of the bladder and bladder urothelial carcinoma, have shown that cystectomy, histological type, histological grade, marital status, year of diagnosis, and gender have been identified as prognostic factors, and PSRCC is a significant independent risk factor for bladder cancer [18, 20]. Wang et al. [8] suggested that age, marital status, AJCC stage, and cystectomy are significant independent risk factors for PSRCC patients. One retrospective analysis for 45 patients from 1981–2008 years also demonstrated that tumor stage and high levels of carcinoembryonic antigen were independent risk factors for tumors [9]. In this study, univariate analyses confirmed that risk factors of PSRCC of the bladder include tumor size (unknown vs. ＜100 mm, HR = 1.834, 95%CI = 1.237∼2.718, *P* = 0.003), M stage (HR = 2.915, 95%CI = 1.832∼4.637, *P* < 0.001), lymph node removed (4 or more regional vs. none, HR = 0.566, 95%CI = 0.384∼0.835, *P* = 0.004), and surgical approach (TURB vs. none, HR = 0.226, 95%CI = 0.107∼0.477, *P* < 0.001; partial cystectomy vs. none, HR = 0.111, 95%CI = 0.042∼0.295, *P* < 0.001; radical cystectomy with reconstruction vs. none, HR = 0.155, 95%CI = 0.072∼0.335, *P* < 0.001; pelvic exenteration vs. none, HR = 0.129, 95%CI = 0.058∼0.289, *P* < 0.001; and other vs. none, HR = 0.138, 95%CI = 0.046∼0.419, *P* < 0.001). However, multivariate analyses showed independent risk factors only include T stage (T3 vs. T1, HR = 4.306, 95%CI = 1.770∼10.478, *P* = 0.001; T4 vs. T1, HR = 2.765, 95%CI = 1.218∼6.277, *P* = 0.015), M stage (HR = 2.343, 95%CI = 1.334∼4.118, *P* = 0.003), lymph node removed (4 or more regional vs. none, HR = 0.477, 95%CI = 0.247∼0.922, *P* = 0.028), and surgical approach (TURB vs. none, HR = 0.255, 95%CI = 0.109∼0.601, *P* = 0.002; partial cystectomy vs. none, HR = 0.125, 95%CI = 0.040∼0.389, *P* < 0.001; radical cystectomy with reconstruction vs. none, HR = 0.193, 95%CI = 0.080∼0.467, *P* < 0.001; pelvic exenteration vs. none, HR = 0.132, 95%CI = 0.049∼0.354, *P* < 0.001; and other vs. none, HR = 0.129, 95%CI = 0.039∼0.424, *P* = 0.001) (Table 2). A previous study has also demonstrated that a significant OS (HR = 0.233, 95CI = 0.107∼0.504, *P* < 0.001) benefits from cystectomy and pelvic lymph node dissection for PSRCC compared with patients undergoing cystectomy only [21]. Data from our study and previous studies proved that the AJCC stage and surgical treatment were independent risk factors for PSRCC. However, our study did not show that age, year of diagnosis, and histological grade are prognostic factors.

However, there are no detailed uniform criteria due to the rarity of the tumor and the lack of clinical trials. Surgery operation and lymph nodes removal are considered protective prognostic factors in prolonged patients' survival. Alradhi et al. [22] reported that surgery served as a significant independent protective factor for PSRCC survival. However, whether surgery should be the most appropriate surgical modality was not further analyzed. In our study, the most common surgery for PSRCC was TURB (49, 31.2%), followed by radical cystectomy with reconstruction (42, 26.8%). Due to the infiltrative pattern of growth and the early propensity of metastasis, nevertheless, certain scholars [23, 24] reported that TURB and partial cystectomy carry the risk of tumor recurrence. Therefore, radical cystectomy appears to be the treatment of first choice [25–27]. According to the CSS curve, we know the survival time is the shortest for unoperated patients, partial cystectomy is the highest, and other surgical treatments are close (*P* = 0.001). In conclusion, it has been found that surgery operation has significantly improved the survival time, so surgery is the main method for PSRCC of the bladder. Recently, 70% patients were reportedly treated with surgery [28]. The number of patients with surgery (146, 93.0%) in the present study was higher than the above values, suggesting that clinicians already have more knowledge of this disease and have attracted increasing attention for surgery.

Given that up to 115 (73.2%) patients were not employing radical cystectomy with reconstruction, their treatments were oppositely prudent and might cause a worse prognosis. We gave some explanation for the condition. Firstly, patients of ≥60 years were observed in 61.8% in our study, and some of them could not undergo radical cystectomy with reconstruction due to their poor health condition. Additionally, for patients with metastasis, losing the optimal opportunities for therapy, they may be considered for palliative treatment rather than radical cystectomy with reconstruction. Finally, muscle-invasive bladder cancer is usually treated with cystectomy, radiotherapy, or systemic chemotherapy. Systemic chemotherapy could cure advanced cancer. In parallel, some recent studies demonstrated that adjuvant chemotherapy may be beneficial for PSRCC [29, 30]. Intravesical chemotherapy has been deemed as the standard treatment option for muscle-invasive bladder cancer patients after receiving TURBT, which could prevent tumor relapse, inhibit tumor growth, and prolong patient survival [31, 32]. We suggested that once PSRCC was considered by biopsy, the combination of advanced therapy should be taken into account.

Although the clinicopathological features and survival outcomes of PSRCC of the bladder were updated based on recent data, the results of our study need to be interpreted with prudery in consideration of several limitations. First, this was a retrospective review in nature. In addition, detailed therapeutic information is lacking, such as radiotherapy and chemotherapy. Future research should aim to obtain information related to radiotherapy and chemotherapy.

## 5. Conclusions

PSRCC of the bladder is a malignant urinary bladder tumor, with a high degree of malignancy and a poor prognosis. Therefore, PSRCC is discovered at a late stage. However, it is characterized by a low risk of lymph node metastases and distant metastases. TURB and radical cystectomy with reconstruction appear to provide a better outcome.

## Figures and Tables

**Figure 1:** Kaplan–Meier survival curves for OS of the entire cohort (a), Kaplan–Meier survival curves for CSS of the entire cohort (b).

**Figure 2:** Kaplan–Meier survival curves for CSS by subgroups of AJCC stage (a), N stage (b), M stage (c), tumor size (d), surgery (e), and lymph nodes removed (f).

**Table 1:** Baseline demographic and clinicopathologic characteristics for PSRCC patients.

Variables	N	N%
Gender		
Female	43	27.4
Male	114	72.6

Age, y		
<60	60	38.2
≥60	97	61.8

Race		
White	133	84.7
Black	16	10.2
Other	8	5.1

AJCC 6th stage		
I	17	10.8
II	34	21.7
III	33	21.0
IV	73	46.5

AJCC 6th T stage		
T1	19	12.1
T2	42	26.8
T3	38	24.2
T4	58	36.9

AJCC 6th N stage		
N0	98	62.4
None N0	59	37.6

AJCC 6th M stage		
M0	130	82.8
M1	27	17.2

Histologic grade		
<IV	108	68.8
IV	49	31.2

Tumor size, mm		
<100	74	47.1
100∼200	8	5.1
Unknown	75	47.8

Year of diagnosis		
2004∼2009	76	48.4
2010∼2015	81	51.6

Surgery		
None	11	7.0
TURB	49	31.2
Partial cystectomy	12	7.6
Radical cystectomy + reconstruction	42	26.8
Pelvic exenteration	34	21.7
Other	9	5.7

Lymph nodes removed		
None	82	52.2
1 to 3 regional	3	1.9
4 or more regional	72	45.9

**Table 2:** Univariate and multivariable analyses of prognostic factors for PSRCC patients.

Variables	Univariate analysis			Multivariate analysis		
	HR	95%CI	*P* value	HR	95%CI	*P* value
Gender						
Female	Reference					
Male	0.745	0.498∼1.116	0.153			

Age, y						
<60	Reference					
≥60	0.857	0.586∼1.253	0.425			

Race						
White	Reference					
Black	1.550	0.864∼2.782	0.142			
Other	0.795	0.323∼1.961	0.619			

AJCC 6th stage						
I	Reference					
II	1.395	0.590∼3.301	0.448			
III	1.900	0.814∼4.437	0.138			
IV	2.836	1.286∼6.254	0.010			

AJCC 6th T stage						
T1	Reference			Reference		
T2	1.349	0.636∼2.861	0.435	1.623	0.744∼3.541	0.224
T3	1.785	0.845∼3.772	0.129	4.306	1.770∼10.478	0.001
T4	1.796	0.869∼3.711	0.114	2.765	1.218∼6.277	0.015

AJCC 6th N stage						
N0	Reference			Reference		
None N0	1.339	0.910∼1.971	0.139	1.275	0.772∼2.108	0.343

AJCC 6th M stage						
M0	Reference			Reference		
M1	2.915	1.832∼4.637	＜0.001	2.343	1.334∼4.118	0.003

Histologic grade						
≤III	Reference			Reference		
IV	0.750	0.490∼1.148	0.185	0.996	0.618∼1.603	0.986

Tumor size, mm						
<100	Reference			Reference		
100∼200	1.962	0.834∼4.619	0.123	1.324	0.516∼3.398	0.559
Unknown	1.834	1.237∼2.718	0.003	1.268	0.802∼2.004	0.310

Year of diagnosis						
2004∼2009	Reference					
2010∼2015	0.875	0.599∼1.276	0.487			

Surgery						
None	Reference			Reference		
TURB	0.226	0.107∼0.477	＜0.001	0.255	0.109∼0.601	0.002
Partial cystectomy	0.111	0.042∼0.295	＜0.001	0.125	0.040∼0.389	＜0.001
Radical cystectomy	0.155	0.072∼0.335	＜0.001	0.193	0.080∼0.467	＜0.001
Pelvic exenteration	0.129	0.058∼0.289	＜0.001	0.132	0.049∼0.354	＜0.001
Other	0.138	0.046∼0.419	＜0.001	0.129	0.039∼0.424	0.001

Lymph nodes removed						
None	Reference			Reference		
1 to 3 regional	1.494	0.467∼4.778	0.499	0.683	0.179∼2.615	0.578
4 or more regional	0.566	0.384∼0.835	0.004	0.477	0.247∼0.922	0.028

## Data Availability

All data that support the findings of this study are openly available in the SEER database from SEER stat v.8.3.8 software.
